# The Effect of Social Stress on Chronic Pain Perception in Female and Male Mice

**DOI:** 10.1371/journal.pone.0047218

**Published:** 2012-10-17

**Authors:** Marjan Aghajani, Mohammad Reza Vaez Mahdavi, Mohsen Khalili Najafabadi, Tooba Ghazanfari

**Affiliations:** 1 Department of Physiology, Faculty of Medical Sciences, Shahed University, Tehran, Iran; 2 Equity and Health Research Department, Shahed University, Tehran, Iran; 3 Department of Immunology, Faculty of Medical Sciences, Shahed University, Tehran, Iran; Northwestern University, United States of America

## Abstract

The current investigations on social stress primarily point to the negative health consequences of being in a stressful social hierarchy. The repetitive nature of such stressors seems to affect behavioral response to pain both in rodents and humans. Moreover, a large discrepancy in the possibility of social stresses affecting pain perception in the two genders exists. The present study examined the effect of chronic social stress on nociceptive responses of both sexes by implementing of food deprivation, food intake inequality and unstable social status (cage-mate change every 3 days) for a period of 14 days in 96 Balb/c mice. In this regard we injected 20 µl formalin 2% into the plantar surface of hind paw at the end of stress period and scored pain behaviors of all subjects, then serum concentrations of proinflammatory cytokines were measured. Our results showed that there was significant difference in chronic phase of formalin test following implementation of food deprivation and inequality (P<0.05) as compared to control group, so that pain perception was decreased considerably and this decline in inequality exposed subjects was well above isolated ones (P<0.05); whereas unstable social situation did not affect pain perception. Moreover, IL-1 and IL-6 concentrations in serum of stressed mice of both genders were well above control group (p<0.05). Finally, despite chronic pain perception in control and unstable male subjects was larger than females; the decrease of chronic pain perception in male stressed animals (poverty and inequality experienced subjects) was much more than stressed females. These results revealed that although food deprivation and social inequality can induce hypoalgesia, some socioeconomic situations like social instability don't affect pain sensation, whereas there were similar increases of proinflammatory cytokines level in all socially stressed subjects. In addition, males display larger hypoalgesic responses to inequality as compared with females.

## Introduction

Health is not just the outcome of genetic or biological processes but is also influenced by the social and economic conditions in which we live. These influences have become known as the ‘social determinants of health’. Inequalities in social conditions give rise to unequal and unjust health outcomes for different social groups [1]. Poverty and social inequality can be intrinsically alienating and distressing, and of particular concern are the direct and indirect effects of poverty on the development and maintenance of emotional, behavioral and psychological problems [2], [3]. Pain is an important sensorial modality with an elevated degree of complexity and subjectivity that involves not only the transduction of noxious stimuli, but also cognitive and emotional features [4], [5]. Several studies have shown the association of the social stresses with the experience of pain [6]–[8]. As in some experiments on animal species, increase in nociceptive thresholds (hypoalgesia) has been found after exposure to social stressors [9]. Nevertheless, other studies have reported that repeated exposure to such stressors can potentiate acute pain perception in humans and animals [10]–[14]. It has been shown both short-term and intermittent food deprivation diminishes acute nociception in laboratory rodents. However, neither prolonged dietary restriction effects nor prolonged pain has received as much attention [15]. Numerous animal models exist for the exploration of mechanism(s) and mediators of persistent pain in particular [16] and such studies in rodents addressing the link between the pain and social stresses are likely to be relevant in humans [17].

Until a few years ago, a large majority of studies used the terms “sex” and “gender” interchangeably. However, an important distinction has been made between the 2 terms: “sex” refers to biological differences between women and men according to their reproductive organs, whereas “gender” refers to a broader and more complex psychological, environmental, socio-cultural, and political framework that encompasses the characteristics ascribed to each sex that are generally accepted and influenced by society (gender role) [18]. Over the years, laboratory and human research has focused on the biological factors that could potentially mediate gender-related differences in pain responses. The role of psychological and social determinants has also been amply investigated [18]–[21]. Sociopsychological explanations for this gender pattern have focused on the greater exposure of women to psychosocial adversity, on women's reporting a variety of recurrent pains than men, as well as differences in responses to stress, which in turn reflect gender differences in role expectations [22].

Thus, the first aim of the present study was to investigate the impact of social stresses on chronic pain perception. Our previous reports provide an impetus that animals as well as humans sense differences in social situations via a bio-psycho-neuro-social phenomenon [23], [24]; in the present study we investigated whether behavioral response to pain could be modulated after implementing different kinds of social stressors. Since recent researches indicate that nervous systems of males and females differently process and react to pain [25], another objective of our study was to evaluate the role of various social factors that may contribute to gender differences in pain sensitivity in laboratory animals.

## Experimental Procedures

### 2.1. Animal model and experimental protocol

96 naive, adult male and female inbred mice of the Balb/c strain (aged 8–10 weeks) were the experimental subjects which were purchased from the Pastour Institute (Karaj, Iran). Ambient temperature was maintained between 22 and 24°C, and the vivarium was maintained under a 12∶12 h light/dark cycle. On arrival, the subjects of each gender were weighted and then randomly assigned to six experimental groups comprising each of eight mice (totally 12 groups). Before the study, the mice were assimilated into the new home for two weeks (there were placed 2 mice of same genders per cage) with no limitation for food (rodent laboratory chow (Daam and Toyur Food Co.) containing by weight: 23.4% protein, 4.5% fat,5% fiber, 7.3% ash, 50% utilizable carbohydrate, and vitamins) and water. Food intake was measured daily and the obtained average amount of ad libitum food consumption was 4.5 gram/day for each mouse. Twelve groups of both genders were set in two rooms: eight groups in one and the remainder in another (isolated) room. After two weeks of assimilating period, three conditions consisting of different social situations [food deprivation, affliction of inequality in food deprived animals (encountering with groups that had free access to diet) and cage-mate change (unstable social status)] were applied to below groups during further 2 weeks:

#### 1. Control group

This group had free access to diet without any deprivation, inequality and change of cage-mate.

#### 2. Food Deprivation (See) group (FD+See)

According to definition of Van Haasteren [26] each mouse in this group received one third (1.5 gram/day) of their normal daily food intake between 09:00 and 11:00 h, and experienced food inequality by sensing that other animals were feeding and smelling food odor, but without any cage-mate change.

#### 3. Food Deprivation (Isolated) group (FD+Isolate)

As same as second group each mouse received 1.5 gr/day food but without experience of social instability (cage-mate change) and any inequality as they were placed in isolated room.

#### 4. Food Deprivation plus Cage-mate Change (See) group (FD+See+CC)

As well as food deprivation and inequality, these animals experienced social instability (cage-mate change every 3 days).

#### 5. Food Deprivation plus Cage-mate Change (Isolated) group (FD+Isolate+CC)

They had similar condition like the fourth group but no experience of food inequality (This group as same as third group were placed in isolated room).

#### 6. Cage-mate Change group (CC)

These animals just faced with social instability (cage-mate change every 3 days) and there was no experience of food deprivation and inequality. In this unstable paradigm [27], one of two mice from each cage was swiped and introduced to another cage in which another resident mouse had experienced this change 3 days ago (such social instability paradigm was also performed in groups 4 and 5).

24 hours after implementing these social stressors (i.e. at day 15 of the study), the animals were weighted again and then they underwent pain assessment which is described in the following section.

It should be noted that food deprivation induces states distinct from physiological situation of caloric restriction [15]. At the end of experiments, the animals were anesthetized and their cardiac blood was collected [28] in order to further investigation about changes of proinflammatory cytokines that will clarify to which extent the observed changes in pain perceptions are attributable to social stresses (it should be noted that we used Balb/c Strain because of their similarity in genetic, just for assessing the effects of social stress on immunological factors [29]), and then they were perished by the high dose of anesthetic agent. The experimental protocols and procedures described in this research were approved by Institutional Animal Care and Use Committee (IACUC) at the Medical University of Shahed (Iran) and complied with the European Communities Council Directive of 24 November 1986 (86/609/EEC). Moreover, all experiments followed the Guidelines on Ethical Standards for Investigation of Experimental Pain in Animals to minimize animal suffering and to use only the number of animals necessary to produce reliable scientific data [30]. Finally, we decided not to determine the phase of the estrous cycle in females because two studies showed that there is no difference in nociceptive responses to the formalin test during these stages [31], [32].

### 2.2. Nociceptive assay

Experiments took place between 12:00 and 16:00. 20 µl of 2% formalin was injected into the plantar surface of the right hind-paw. Mice were standing on a glass floor within Plexiglas observation cylinders (25 cm diameter; 22.5 cm high) and habituated to these cylinders to be tested concurrently for 30 minutes before the formalin injection. Then they were briefly removed, injected and replaced in the cylinder and their pain response was scored every 15 second for 60 minute according to below sampled scales:

0- ***no pain*** **:** normal weight born on injected paw
1- ***favoring*** **:** injected paw in contact with the floor, but full weight not on the paw
2- ***lifting*** **:** injected paw elevated
3- ***licking*** **:** licking or biting the injected paw

The observational period was divided into 20 blocks of 3 minutes each (at which we firstly calculated the mean pain score of each minute and then the mean pain score of each block), so we had a biphasic diagram at which a first peak of behavioral response to pain (typically licking behavior of the formalin-injected paw) during the first 6 minute interval reflected the behavioral response to acute pain; whereas the second part of the curve represented a persistent pain (the average scale from minutes 15 to 35 was considered as chronic phase [33]). In between the two curves, there was an inter-phase in which paw-licking behavior was almost reduced to zero [34].

### 2.3. Immunological assay

After formalin test, mice were anesthetized slightly with ether and then while we sensed heart beats from apex, blood samples were obtained from ventricle. For measurement of cytokine concentrations clotted blood samples were centrifuged immediately at 3000 rpm for 10 minutes and serums stored at −70°C. Circulating immunoreactive IL-6 and IL-1 levels were measured using commercially available quantitative enzyme-linked immunosorbent assays (R&D Systems Europe, Abingdon, UK) [35]. The assays did not measure biological activity of the cytokines. Standard sensivity assays were used and the manufacturers reported the sensivity thresholds in serum as 0.7 pg/ml and 1.5 pg/ml for IL-6 and IL-1, respectively. All measurements were made by a single trained individual to avoid interobserver variation.

### 2.4. Statistical analysis

Statistical analyses were performed using the Sigma Stat software (Systat Sofware, Inc., Point Richmond, CA, USA). Analyses included Mann-Whitney U test for non-parametric data (gender differences), two-way ANOVA test (the effect of each social stressor on the mean nociceptive score in each phase (I, interphase, II) of the formalin test) and one-way ANOVA test (statistical significance for cytokines concentrations) for multiple comparisons, followed by the post hoc Tukey–Kramer test for parametric distribution. Additionally, the results of pain behaviors after formalin injection were analyzed with a one-way ANOVA for repeated measures (10 blocks) to test difference between all blocks in each group. A significance level of P<0.05 was used in all cases. Data are presented in the text and in all figures as means ± SEM.

## Results

### 3.1. Body weight

Control and all experimental animals were similar in body weight before procedure. As shown in **Figure 1**, body weight of groups which experienced food poverty merely or coincided with food inequality (with or without cage-mate change) for 14 days, was less than their initial body weight (p<0.05), and there was no significant difference between male and females in this regard. Unstable social status resulted in weight loss but this decline was not considerable both in males and females (male: p = 0.081; female p = 0.054); this served to indicate that just food poverty and inequality paradigm has caused obvious weight loss.

**Figure 1:** Body weight changes in male mice exposed to chronic psychosocial stress. Implementing food poverty merely or coincided with food inequality (with or without cage-mate change) have caused significant decrease in body weight of both males and females (there is no difference between these two genders). FD+See: Food Deprived and inequality experienced group, FD+Isolate: Food Deprived group without inequitable situation, FD+CC+See: Food Deprived group which also experienced inequality and cage-mate change simultaneously, FD+CC+Isolate: Food Deprived and cage-mate change experienced group without inequitable situation, CC = the group which just experienced cage-mate change. *p<0.05: beginning of study vs. end of chronic social stress (Values are means ± SEM; n = 6–8 animals in each group).

### 3.2. Comparison of chronic pain perception between control and socially stressed males and females

A repeated measure one-way ANOVA analysis detected the characteristic biphasic curve of the formalin-induced behavioral response in control groups. Classically, a first peak of Licking behavior during the first 6 minute block reflects the behavioral response to acute pain, whereas the second part of the curve represents persistent (chronic) pain. Interestingly, this biphasic response was not observed in animals which underwent food deprivation merely or coincided with food inequality (**Figures 2** **–** **5**); according to these findings pain behavior had no increase at the second phase of formalin test in food deprived and inequality experienced animals which showed a significant effect of these social stressors on creation of hypoalgesia (p<0.05). For confirmation this point, we used repeated measurement one-way ANOVA in order to compare 3-min blocks in a group; so it revealed there was no significant difference between 3-min blocks of formalin test's second phase in food deprived and inequality experienced mice (groups 2 to 5). In animals which just experienced cage-mate change (unstable social status) a biphasic curve after injection of formalin was created as same as control groups; representing that chronic pain perception was not affected by this type of social stressor (**Figure 6**).

**Figure 2:** Effect of food deprivation and inequality without cage-mate change on pain behavior during the formalin test. The observation period is divided into 20 blocks of 3 minutes each. Unlike control male and female subjects, biphasic curve was not observed in animals which underwent food deprivation and inequality simultaneously (Data are means ± SEM, females; Control and FD+See: n = 8, males; Control: n = 7 and FD+See: n = 6).

**Figure 3:** Effect of food deprivation merely, without inequality and cage-mate change on pain behavior during the formalin test. The observation period is divided into 20 blocks of 3 minutes each. In all stressed animals as compared to controls, pain behaviors did not appear in chronic phase of formalin test (Data are means ± SEM, females; Control and FD+Isolate: n = 8, males; Control and FD+Isolate: n = 7).

**Figure 4:** Effect of food deprivation, inequality and cage-mate change on pain behavior during the formalin test. The observation period is divided into 20 blocks of 3 minutes each. In all stressed animals as compared to controls, pain behaviors did not appear in chronic phase of formalin test (Data are means ± SEM, females; Control and FD+See+CC: n = 8, males; Control and FD+See+CC: n = 7).

**Figure 5:** Effect of food deprivation and cage-mate change without food inequality on pain behavior during the formalin test. The observation period is divided into 20 blocks of 3 minutes each. Pain behavior of stressed animals was not revealed during the chronic phase of formalin test as compared to controls (Data are means ± SEM, females; Control and FD+Isolate+CC: n = 8, males; Control and FD+Isolate+CC: n = 7).

**Figure 6:** Effect of cage-mate change merely without food deprivation and inequality on pain behavior during the formalin test. The observation period is divided into 20 blocks of 3 minutes each. Implementing cage-mate change merely did not affect pain behaviors during the chronic phase of formalin test as same as controls (Data are means ± SEM, females; Control and FD+Isolate+CC: n = 8, males; Control and FD+Isolate+CC: n = 7).

As shown in **Figure 7**, chronic pain perception both in males and females not only was affected by food deprivation but also by food inequality; expressing that implementing of such stressors has caused significant decrease of chronic pain sensation (hypoalgesia) compared with control group (p<0.001).This decline in food deprived mice along with inequitable situation was greater than isolated food deprived animals, ((FD (See) vs FD (Iso): p<0.001 and FD+CC (See) groups vs FD+CC (Iso) groups: p<0.001). However, as mentioned before, the second phase response in 6^th^ group (merely experienced unstable situation) did not show significant difference with control group (male: p = p = 0.932; female: p = 0.98).

**Figure 7:** Effect of different social stressors on second-phase responses to formalin. The score of pain behaviors between 15 and 35 min after formalin injection is plotted, along with the standard error of the mean (n = 6–8 in each group). As it is obvious, unlike food poverty and inequality, cage-mate change did not influence chronic pain perception as like controls. Moreover, food deprived and inequality experienced males perceive pain as less as females. *p<0.05: significant difference between stressed and controls of females. ^#^p<0.05: significant difference between stressed and controls of males. ^&^ p<0.05: significant difference between males and females.

### 3.3. Comparison of chronic pain perception between males and females

As expected (**Figure 7**), a significant main effect of gender emerged (p = 0.032) reflecting the generally greater pain perception exhibited by control males relative to control females. Moreover, pain perception of male subjects which just experienced unstable situation, was well above in comparison with similar group of females (p = 0.013). Comparison of male and females of food deprived animals which experienced inequitable situation with or without cagemate change, showed males were hypoalgesic than females (FD+See and FD+CC+See animals: p<0.001); however, there was no significant difference between isolated subjects which underwent food poverty with or without cagemate change (FD+Isolated animals: p = 0.16, FD+CC+Isolted animals: p = 0.308). **Figure 8** reveals that the level of pain decrease toward control subjects, in food deprived and inequality experienced males is well above its decrease in similar stressed females (p<0.05).

**Figure 8:** The level of pain decrease in socially stressed animals toward control groups. It is clear that male subjects which experienced food inequality, revealed further hypoalgesic response as compared to females. Data are means ± SEM. *p<0.05: significant difference between stressed and controls of females. ^#^p<0.05: significant difference between stressed and controls of males.

### 3.4. Comparison of serum cytokines levels between control and experimental groups

As shown in **Figure 9**, evaluation of IL-6 concentration in serum of experimental subjects both in females and males showed IL-6 levels in all animals which underwent food deprivation, food inequality and cage mate change have increased significantly as regards control mice (p<0.05) and this increase in males and females which experienced all three stresses is well above other stressed animals; although this difference toward some of these groups is not significant. In addition, beside high levels of IL-1 concentration (**Figure 10**) in stressed mice as compared to controls (p<0.05); IL-1 concentration in serum of food deprived animals which experienced unstable social status and unequality simultaneously, was also more than other stressed animals of both genders (p<0.05).

**Figure 9:** Effect of of different social stressors on serum concentration of proinflammatory cytokines (Interleukin-6) in mice. Data are means ± SEM. *p<0.05: significant difference between stressed and controls of females. ^#^p<0.05: significant difference between stressed and controls of males.

**Figure 10:** Effect of of different social stressors on serum concentration of proinflammatory cytokines (Interleukin-1) in mice. Data are means ± SEM. *p<0.05: significant difference between stressed and controls of females. ^#^p<0.05: significant difference between stressed and controls of males.

## Discussion

The purpose of this study was to investigate how the male and female animals differ in their experience of experimental chronic pain and whether long-term social stresses differentially affect this response. To achieve these goals, adult male and female mice were subjected to a model of chronic social stress which offers the opportunity to investigate about differences of pain perception in association with social stresses and gender. We found that, all male and female subjects which underwent food poverty and inequality with or without social instability were hypoalgesic in chronic phase of formalin test as compared to control animals. However, social instability merely didn't affect chronic pain perception after subcutaneous injection of 2% formalin in both genders. In addition, this hypoalgesic response in food deprived and inequality experienced males was well above females.

### 4.1. Effects of chronic social stresses on chronic pain perception in both genders

Pain research has shown that (1) not all noxious stimuli are processed centrally or peripherally in the same way and (2) not all aversive stimuli are capable of eliciting an analgesic response and can in fact elicit a hyperalgesic response [36]. Studies have shown that being in chronic pain rather than acute pain express elevated pain behaviors in the presence of an aversive stimulus [37]. However, little has been previously reported about the effects of chronic social stress on persistent pain, despite different studies have shown the prevalence of pain in people who experience a long term period of stress, is much less [34], [38], [39]. Pain can be characterized by its duration (from momentary to chronic), location (e.g., muscle, viscera), or cause (e.g., nerve injury, inflammation). Characterization of pain by duration may be arbitrary (i.e., when does pain become chronic?), but is useful because most significant human pain conditions are long-lasting, whether referred to as persistent or chronic [16]. The majority of experimental pain results obtained in animals are consistent with those obtained in humans. These findings have been observed using various experimental tests and nociceptive modalities, but have often been investigated in the formalin test [32], [40], [41]. Rodent hind paw inflammation is a commonly used model of persistent inflammatory pain in which hind paw injection of formalin or capsaicin is used to assess intense, short-lasting (minutes to tens of minutes) persistent pain [16]. The results of this study are consistent with the notion that even food poverty and inquality can be stressful, in turn provoking a physiological reaction akin to that which occurs upon perception of a physical threat [42] one component of which can be hypoalgesia. Anatomical, pharmacological and behavioral evidence from stressed-induced analgesia studies revealed that amygdale, periaqueductal grey (PAG) and rostral ventromedial medulla (RVM) as critical structures, contribute to descending inhibitory pain pathways and lesions of these structures attenuate the conditioned stressed-induced analgesia response which can be mediated by opioid receptors [38], [42]. Opioids hypoalgesic effects are particularly prominent in inflammatory conditions [43]. Implementing of food deprivation and inequality for a period of two weeks resulted in significant decrease in body weight, which was more pronounced in female mice; so it seems that such weight loss can be in accordance with limitation of calorie during deprivation that can lead to a potentiated hypoalgesic response [44]. Studies of malnourished children have shown that Protein-Energy Malnutrition may lead to oxidative stress, which can lead to increased activity of proinflammatory cytokines [45], this finding is in accordance with our following researches about increase of serum proinflammatory cytokines concentration (IL-6, IL-1) beside oxidative stress markers (data has not been published) such as MDA (Malon-Di-Aldehyde), especially in food deprived and inequality undergoing mice. It seems more probably that attenuated sensivity of immune cells to glucocorticoids [46] after implementing mentioned social stressors have caused extra levels of proinflammatory cytokines. So, inflammation of peripheral tissue as well as increasing the number of nociceptor endings and disrupting the peri-neural barrier which facilitates the access of opioid agonists to their receptors [47], leads to increased synthesis and axonal transport of opioid receptors in DRG neurons, resulting in their up-regulation and enhanced G-protein coupling at peripheral nerve terminals [48].

The body produces its own powerful pain-modulating neurotransmitters. It is stated chronic stressors combined with a diet low in protein, can create deficiencies in the three most critical of these pain-modulators: serotonin, gamma-amino-butyric acid (GABA), and endorphin. In Practical Pain Management, the use of diet and amino acid supplementation in promoting optimal levels of serotonin, GABA and the endogenous opiates have been discussed, as it was emphasized that if adequate protein is consumed, endorphin levels may remain high enough to effectively modulate pain [49], [50]. However in present study we took in consideration that hypoalgesic response after food deprivation (which may lead to katabolism and decrease of body's total protein) is likely related to activation of endogenous opiates, so further investigation are needed to explain this contradiction.

Stress can affect pain perception differentially, as accession of hypealgesia or hopoalgesia depends on the type of stressor as well as its intensity and duration [51]. It was stated that highly unstable situation does not predict elevated basal cortisol concentrations in an individual [52]. As we saw in our study, pain behavior in unstable group (cage-mate changed) did not differ from control animals; so we can presume that our social instability paradigm did not release opioids to create stress-induced hypoalgesia, despite serum concentrations of IL-1 and IL-6 have increased at this group and it seems more probably that hypoalgesic response after food deprivation and inequality is regulated via pathways different from proinflammatory cytokines; so further mechanistic invesigations are needed to reveal what is the cause of this contradiction.

### 4.2. Gender differnces in chronic pain perception after implementing social stresses

Clinically it is well documented that women are more likely than men to report a variety of recurrent pains which are often described as being more severe and frequent compared to men [53]. Therefore, numerous laboratory studies have been conducted to try to understand the mechanisms underlying these difference [25], [53], [54]. However, very few studies have investigated gender differences in chronic pain models such as nerve injury and persistent inflammation [19]. Concerning gender differences, male rodents exhibit larger hypoalgesic responses to environmental stress - a natural trigger that serves to activate the same descending analgesia pathways that are acted upon by centrally acting opiate drugs. Such findings suggest that both ascending and descending pathways involved in the experience of pain are influenced by hormonal or other gender-related factors [22]. We observed herein that male mice display significantly more hypoalgesia than females following food deprivation and inequality and it seems males are more prone to adverse effect of social inequality. The reasons for these discrepancies remain unknown, but the possibility of hormonal factors to affect the magnitude of analgesic responses should not be overlooked. The potential importance of gonadal hormones in accounting for gender differences in opioid-induced antinociception has been examined in numerous investigations [55]. Although there are discrepancies in the literature, a number of reports suggest that gonadal hormones play a clear role in opioid antinociception [32], [56]. Indeed it is stated that gonadal steroid hormone binding sites are ubiquitously distributed throughout central nervous system regions involved in pain perception and pain inhibition, such as the periaqueductal gray, rostroventral medulla, and spinal cord dorsal horn [22]. While the reasons for a lack of an effect of menstrual cycle phase on gender differences in pain sensitivity are not known, one possibility relates to a putative threshold effect of gonadal hormones on pain sensitivity. For example, even in the early follicular phase of the menstrual cycle when estrogen and progesterone are at their lowest, women still exhibit significantly greater hormone levels than men [57]. Despite some studies have shown estrogens seem to play a role in inducing hyperalgesia and pain [58], [59], analgesic effects of estrogen and progesterone in animals have been documented [60], but consistency in the pattern and direction of the relationship between hormones and nociception is lacking and underlying mechanisms have yet to be elucidated [57], [61]. Accordingly, it seems high levels of these gonadal hormones in females as compared to males can be a reason for high persistent pain perception in control females in our study; however, since it is shown that the largest effects of esterogen and/or progestrone occur during the interphase of formalin test [40], we can suggest that the discrepancy between food deprived and inequality experienced males and females in persistent pain response can be influenced by several biological (genes and hormones) and other confounding socio-environmental factors, not just by gonadal hormones diversity.

Consequently, the present results suggest that deprivation and social inequality affect persistent pain perception and are probably involved in the activation of endogenous analgesic systems in mice, despite unstable social status doesn't put any effect on pain response and modulated it via pathways different from proinflammatory cytokines; so understanding the mechanisms is crucial to facilitate our knowledge about how various social and environmental factors can affect pain perception. Moreover, results from this study should help pave the way to a better understanding of gender differences in pain processing.
